# Diagnosis of Idiopathic Premature Ovarian Failure by Color Doppler Ultrasound under the Intelligent Segmentation Algorithm

**DOI:** 10.1155/2022/2645607

**Published:** 2022-05-25

**Authors:** Lanlan Yu, Xiaofeng Qing

**Affiliations:** Department of Gynaecology, The First People's Hospital of Huaihua, Huaihua, 418000 Hunan, China

## Abstract

The aim of this study was to explore the application value of transvaginal color Doppler ultrasound based on the improved mean shift algorithm in the diagnosis of idiopathic premature ovarian failure (POF). In this study, 80 patients with idiopathic POF were selected and included in the experimental group, and 40 volunteers who underwent health examinations during the same period were selected and included in the control group, who underwent transvaginal Doppler ultrasound examination. At the same time, an improved mean shift algorithm was proposed based on artificial intelligence technology and applied to ultrasound image processing. In addition, the ovarian artery parameters of patients were compared in two groups, including peak systolic flow rate (PSV), diastolic flow rate (EDV), resistance index (RI), and pulsatile index (PI). The results showed that the relative difference degree (RDD) of the segmentation results of the algorithm in this study was significantly lower than that of Snake, Live_wire, and the traditional mean shift algorithm, while the relative overlap degree (ROD) and Dice coefficient were opposite, and the differences were significant (*P*<0.05). The mediolateral diameter of control group was 2.87±0.31cm, and the anteroposterior diameter was 1.86±0.28 cm; while those were 2.11±0.36 cm and 1.13±0.34 cm, respectively, in the experimental group, showing significant differences between the groups (*P*<0.05). Of the 80 patients in the experimental group, 132 cases with ovarian arteries were found; among 40 patients in the experimental group, 76 cases were found with ovarian arteries, and the hemodynamic detection rate of the experimental group was significantly lower than that of the control group (*P*<0.05). The ovarian artery parameters PI, RI, and S/D of the experimental group were significantly higher than those of the control group, and the differences were statistically significant (*P*<0.05). The results showed that the segmentation results of the improved algorithm in this study were more superior to the segmentation results of other algorithms. The regional information loss of the segmentation results was not serious, and the resolution was higher and the definition was higher. The transvaginal color Doppler ultrasound based on the artificial intelligence segmentation algorithm can clearly show the functional status and hemodynamics of the patient's ovaries. The ovarian artery parameters PI and RI can be used as specific indicators for evaluating the POF.

## 1. Introduction

Premature ovarian failure (POF) refers to the phenomenon of amenorrhea before the age of 40 caused by ovarian failure [1]. It is characterized by primary or secondary amenorrhea accompanied by increased blood gonadotropin levels and decreased estrogen levels, accompanied by a series of low estrogen symptoms of varying degrees [2, 3]. Idiopathic POF is a kind of secondary amenorrhea with no clear causative factors, and is the most important type of POF, which usually develops in the reproductive age; and clinically, gradual or progressive menstruation occurs, amenorrhea is accompanied by menopausal symptoms such as hot flashes and irritability, and the internal and external reproductive organs are in atrophied state [4–6]. The currently known treatment factors include chromosomal abnormalities, autoimmune diseases, iatrogenic injuries, and viral infections. In addition, age, family history, and multiple ovarian surgeries are high-risk risk factors for POF [7]. The early symptoms of POF can be manifested as oligomenorrhea or frequent menstruation. Typical symptoms include primary amenorrhea, secondary amenorrhea, low estrogen, and infertility. At present, there is no clear method to help patients restore the function of the ovaries, which generally means psychological intervention, drug therapy (estrogen supplementation therapy and progesterone), and traditional Chinese medicine (TCM) treatment [8, 9].

In clinic, doctors can judge whether POF occurs by observing the patient's general development, mental state, intellectual development, and nutritional status. Laboratories can use pregnancy tests, drug withdrawal tests, progesterone tests, and estrogen and progesterone sequential tests [10]. Transvaginal color Doppler ultrasound is a non-invasive examination technique. The probe is closely attached to the cervix and vaginal vault in the vagina. Using high-frequency technology and local magnification function, it can clearly show the changes of cavity anatomy and subtle sound image, making the monitoring image more intuitive, clear, and accurate, and suitable for observing the ovarian, uterine cavity, and other subtle sound image structures. It can display the ovarian size, morphology, cortical and medulla ratio distribution, and the number, size, and dynamic development of follicles [11, 12]. However, ordinary ultrasound images cannot clearly reflect the organs and tissues, which also brings certain difficulties to clinical diagnosis and follow-up treatment. Clinically, the doctor can make a preliminary estimate of the condition through the ultrasound image of the patient, and the edge segmentation of the target lesion is generally manual. This method shows strong subjectivity, is related to the doctor's clinical experience, and has a large workload, which requires detailed optimization of the original ultrasound graphics. The segmentation of medical ultrasound images is very difficult in practice, and there is still no effective segmentation method [13, 14]. Although the traditional threshold segmentation method is very convenient and simple to implement, the inevitable speckle noise and complex texture in ultrasound images make it difficult to obtain satisfactory results. Mean Shift algorithm aims to segment images into regions with semantic meaning, and has been widely used in the field of medical image processing [15].

In summary, the diagnosis and treatment of idiopathic POF is a topic that needs clinical attention at present, and ultrasound imaging technology has strong applicability. Therefore, in this study, 80 idiopathic POF patients were used as the experimental group, and 40 volunteers who underwent health examinations during the same period were used as the blank control group. All of them underwent transvaginal color Doppler ultrasound based on artificial intelligent segmentation algorithm. The ovarian artery parameters, hemodynamics, and the situation of the two groups of patients were compared to comprehensively evaluate the diagnostic value of artificial intelligence algorithm combined with color Doppler ultrasound on idiopathic POF.

## 2. Materials and Methods

### 2.1. Research Objects

In this study, 80 patients with idiopathic POF who were treated in hospital from October 2019 to March 2021 were selected as the research objects (the experimental group). In addition, 40 volunteers who underwent physical examination during the same period were selected as the control group. This study had been approved by ethics committee of hospital. The patient and the family members of all research objects had understood the situation of the study and signed the informed consent forms.

The patients meeting below criteria could be included in the experimental group: patients with amenorrhea more than six times before the age of 40; patients whose serum follicle stimulating hormone was greater than 40 IU/L in more than two examinations; patients who were married; patients with normal menarche and development of secondary sexual characteristics. Patients meeting below criteria had to be excluded: patients with age greater than 40 years old and unmarried patients.

Inclusion criteria in the control group were defined as follows: normal menstrual cycle; seeing a doctor for other reasons; younger than 40 years old; and married patients. The exclusion criteria were given as follows: age greater than 40 years old; unmarried patients; patients with a history of ovariectomy; and patients with uterine fibroids and ovarian cysts.

### 2.2. Doppler Ultrasonography

Color ultrasound diagnostic system was adopted. The probe was 5.5 - 7.5 MHZ, and the fan expansion angle was 120 - 240 degrees. The probe was rotated to the left or right to find the ovary. When the display was clear, it could measure the mediolateral diameter and anteroposterior diameter of the ovary. The color sampling frame was placed on the ovary, the blood flow of the stromal artery in the medulla of the ovary was taken, and 3 ~ 5 cardiac cycles were obtained continuously after getting a satisfactory spectrum. The peak systolic velocity (PSV) and end diastolic velocity (EDV) of the ovarian artery can be measured. In addition, the ultrasonic diagnostic apparatus automatically calculated the resistance index (RI) and pulsatility index (PI).

### 2.3. Improved Mean Shift Algorithm

Mean shift algorithm [16] is a segmentation algorithm based on scatterer analysis. The process of finding the center of the scatterer through continuous iterative calculations and the movement traces during the recording process can achieve filtering and smoothing, area segmentation, or target tracking. Although the mean shift algorithm shows a good segmentation effect for ordinary gray-scale images, the outline is clear, and there are fewer false borders. However, the effect is not ideal when applied directly to ultrasound image segmentation. The traditional mean shift algorithm was compared with the original image. As shown in Figure 1, due to the large or small bandwidth, over-segmentation and loss of information edges were found, and there was a pseudo area in the lower half of the large sphere of the segmentation map in the lower right corner. The size of the threshold for the final merge led to the unsatisfactory results of the segmentation.

In view of this, the image space feature and grayscale feature were added to the segmentation process, and finally the threshold was applied to remove the fragments in the segmented image. The main flow of the algorithm can be shown in Figure 2 below.

The traditional mean shift segmentation algorithm is fixed in terms of bandwidth selection, which makes the window in the moving process and the bandwidth parameters unable to change in real time, which affects the operating efficiency and accuracy. Therefore, the algorithm in this study adopted the following bandwidth selection function [17]:

(1) $$\begin{array}{c} f_{r\left(t\right)}=f_{\max}\left(1-z_{t}e^{-{\left(t-t_{ROI}\right)}^{2}}\right) \end{array}$$

In the equation (1) above, *f*_*r*(*t*)_ represented the grayscale bandwidth, *f*_max_ represented the maximum bandwidth, *t* represented the pixel grayscale, *t*_*ROI*_ referred to the grayscale of the region of interest, and *z*_*t*_ represented the weighting coefficient. Using a larger bandwidth in a dense area and a smaller bandwidth in a sparse area can increase the efficiency and accuracy of the algorithm, and then determine the weighting coefficient. The weighting coefficient would affect the size of the bandwidth. The weighting ratio of the dense texture direction was large, and the bandwidth should be small to prevent loss of details; on the contrary, the bandwidth should be large to avoid over-segmentation. The value of the weighting coefficient can be expressed as follows:

(2) $$\begin{array}{c} z_{t}=\frac{Q_{\max}}{\sum Q_{i}} \end{array}$$

In equation (2) above, *Q*_*i*_ represented the average value of each texture image, and *Q*_max_ represented the maximum value in the feature vector library. At the end of the algorithm, threshold clustering and merging were needed to prevent over-segmentation and make the result more ideal. The equation can be expressed as below equation:

(3) $$\begin{array}{c} \left|p_{i}-p_{j}\right|\leq H \end{array}$$

In the equation (3) above, *p*_*i*_ and *p*_*j*_ denoted two adjacent regions, and *H* was the threshold, whose value was automatically calculated and determined by the image direction texture energy map using the filter operator method. This operation was to merge the two regions in the image where the average difference between the pixel averages of adjacent regions in the image filtered by the mean shift algorithm was less than H, and then merge the non-protruding mode regions near them according to the mode position. After all modes were filtered, the segmentation was completed.

### 2.4. Segmentation Experiment

Introduce active contour model (Snake) [18], interactive segmentation algorithm (Live_wire) [19], and traditional mean shift algorithm were introduced and compared with the improved mean shift algorithm designed in this study.

Relative difference degree (RDD) [20], relative overlap degree (ROD) [21], and Dice coefficient [22] were used to quantitatively analyze the accuracy of segmentation results.

RDD represented the degree of difference between the segmentation result and the actual target, which can be expressed as follows:

(4) $$\begin{array}{c} RDD=\frac{\left|U_{2}\right|-\left|U_{1}\right|}{\left|U_{2}\right|} \end{array}$$

In the equation (4) above, ROD represented the relative degree of overlap between the segmentation result and the actual target, which can be expressed as below equation:

(5) $$\begin{array}{c} ROD=\min\left\{\frac{\left|U_{2}\right|\cap \left|U_{1}\right|}{\left|U_{2}\right|}*\frac{\left|U_{2}\right|\cap \left|U_{1}\right|}{\left|U_{1}\right|}\right\}*100\% \end{array}$$

In equation (5), the Dice coefficient was used to indicate the relative overlap between the segmentation result and the actual target, which can be expressed as follows:

(6) $$\begin{array}{c} Dice=\frac{\left|U_{2}\right|\cap \left|U_{1}\right|}{\left|U_{2}\right|+\left|U_{1}\right|}\times 2 \end{array}$$

In equation above, *U*_2_ represented the actual target, and *U*_1_ represented the segmentation result.

### 2.5. Statistical Methods

The data processing of this study was analyzed by SPSS19.0 version statistical software, the measurement data was expressed by the mean±standard deviation (^−^x±s), and the count data was expressed by the percentage (%). One-way analysis of variance was used for pairwise comparison. The difference was statistically significant at *P*<0.05.

## 3. Results

### 3.1. Analysis on Experimental Results

As shown in Figure 3 below, the RDD of the segmentation results of the algorithm in this study was significantly lower than that of Snake, Live_wire, and the traditional mean shift algorithm, and the differences were statistically significant (*P*<0.05). The ROD and Dice coefficient of the segmentation results of the algorithm in this study were significantly higher than those of Snake, Live_wire, and the traditional mean shift algorithm, and the differences were statistically significant (*P*<0.05).

The segmentation results of the four algorithms for ultrasound images were compared (Figure 4). It can be observed that the segmentation results of the improved algorithm in this study had more advantages compared with the segmentation results of other algorithms. The regional information loss of the algorithm segmentation results in this study was not serious, the resolution was higher, and the definition was higher. The segmentation results of the Snake model and the Live_wire algorithm showed serious loss of detail information. Although the traditional mean shift algorithm retained better segmentation information, the definition was low, and the area information was blurred.

### 3.2. The General Situation of Research Objects in the Experimental Group and the Control Group

Figure 5 showed the general situation of research objects in the experimental group and the control group. It illustrated that the differences in age, height, weight, hypertension, hyperlipidemia, and smoking history of the experimental group and the control group were not statistically significant (*P*>0.05).

### 3.3. Ultrasound Data of a Patient before and after Treatment

Figure 6 showed the case data of a 24-year-old patient. Before treatment, the patient had already experienced symptoms of decreased ovarian function, such as decreased physical strength, decreased sensitivity of the body's various sensory organs, and dry skin. Transvaginal color Doppler ultrasound examination (Figure 6(a)) showed that the endometrium was 0.5 cm thick and was C-shaped. The echo of the right ovary was solid, no follicular echo was seen, and 3 follicular echoes were seen on the side of the left ovary. After treatment, the patient showed increased physical strength, clear ears and eyesight, peace of mind, fair skin, etc. The transvaginal color Doppler ultrasound examination (Figure 6(b)) showed that the endometrial thickness was 0.8 cm, which was C-shaped. There were multiple follicular echoes on the same side of both ovaries, and the largest follicle on the right was 1.8 cm ×1.2 cm.

### 3.4. Comparison of Ovarian Size between Experimental Group and Control Group

Figure 7 showed the comparison of the ovarian size between the experimental group and the control group. The mediolateral diameter of the patients in control group was 2.87±0.31 cm, and the anteroposterior diameter was 1.86±0.28 cm; the mediolateral diameter of the patients in experimental group was 2.11±0.36 cm, and the anteroposterior diameter was 1.13±0.34 cm. It revealed that the mediolateral diameter and anteroposterior diameter of the control group were significantly larger than those of experimental group, and the differences were statistically significant (*P*<0.05).

### 3.5. Hemodynamic Detection Rates in Experimental Group and Control Group

As illustrated in Figures 8, of the 80 patients in the experimental group, 132 ovarian arteries were detected and 28 were not detected; among 40 patients in the control group, 76 ovarian arteries were detected and 4 were not detected. The hemodynamic detection rate of the experimental group (82.5%) was significantly lower than that of the control group (95%), and the difference was statistically significant (*P*<0.05).

### 3.6. Comparison of Ovarian Artery Parameters between the Experimental Group and the Control Group

The ovarian artery parameters were compared between the experimental group and the control group, and the results were given in Figure 9. It showed that the ovarian artery parameters EDV and PSV of the experimental group were significantly lower than those of the control group, and the differences were statistically significant (*P*<0.05). In addition, the ovarian artery parameters PI, RI, and S/D of the experimental group were significantly higher than those of the control group, and the differences were statistically significant (*P*<0.05).

## 4. Discussion

Ovary is an important body organ for women. From menarche to natural menopause, ovary plays a vital role. Generally speaking, women will not have ovarian failure until the age of 45 or even 50. However, some female friends, due to various reasons, lead to the symptoms of POF at the age of less than 40 [23]. Generally speaking, most women have menstrual cramps for the first time since the age of 14, and will experience regular menstruation once a month at the age of 50 or even 55 (except during pregnancy). However, before the age of 40, some women will experience ovarian failure due to depletion of follicles in the ovary or damage caused by some external causes, resulting in menstrual disorders such as menopause or oligomenorrhea. In addition, it is characterized by low estrogen and high gonadotropin. Once this symptom lasts for 4 months, it is considered that POF occurs. POF has become one of the hot spots in the field of gynecology, and its diagnosis and treatment research is very necessary [24, 25]. In this study, 80 idiopathic POF patients were selected as the research objects and set as the experimental group. In addition, 40 volunteers who underwent health checkups during the same period were selected and set as the blank control, which underwent transvaginal color Doppler ultrasound. Based on artificial intelligence technology, an improved mean shift algorithm was proposed and applied to ultrasound image processing. The performance analysis of the algorithm designed in this study found that the RDD of the segmentation result the algorithm used in this study was significantly lower than the Snake, Live_wire, and traditional mean shift algorithm, while the ROD and Dice coefficient were significantly higher than those of other algorithms, showing statistically significant differences (*P*<0.05). Such results are similar to the study of image segmentation algorithm by Brattain et al. [26], which shows that the segmentation results of the ultrasound image of the algorithm in this study are similar to the actual target, and the degree of overlap is better. The display of the ultrasonic image segmentation results of the four algorithms was compared. It revealed that the segmentation results of the improved algorithm in this study showed more advantages compared with the segmentation results of other algorithms. The regional information loss of the algorithm segmentation results in this study was not serious, the resolution was higher, and the definition was higher. Such results are consistent with the findings of the above quantitative data, and both confirm that the image segmentation performance of the algorithm in this study is excellent.

The mediolateral diameter of the patients in control group was 2.87±0.31 cm, and the anteroposterior diameter was 1.86±0.28 cm; the mediolateral diameter of the patients in experimental group was 2.11±0.36 cm, and the anteroposterior diameter was 1.13±0.34 cm, showing statistically significant differences (*P*<0.05). Such results are similar to the findings of Zhang et al. (2022) [27]. Ovarian volume is closely related to the size of the follicle. The blood hormone level can be understood by measuring the size of the follicle. This result showed that compared with normal people, the ovaries of patients with idiopathic premature ovarian failure will have obvious atrophy, and the smaller size of the ovary and the decrease of reproductive hormones are the important characteristics of judging premature ovarian failure. Ovarian artery is an important blood vessel for follicular development. Ovarian artery resistance decreases, diastolic flow rate increases, and ovarian blood perfusion is good when the frequency spectrum shows obvious characteristics of high-speed and low-resistance, which is conducive to follicular development and easy to conceive. If there is no abundant diastolic blood flow in the ovaries during follicular development, it indicates that the follicles cannot develop normally [28]. It was found in this study that among 80 patients in the experimental group, 132 ovarian arteries were detected and 28 were not detected; among 40 patients in the control group, 76 ovarian arteries were detected and 4 were not detected. Therefore, the hemodynamic detection rate of the experimental group was significantly lower than that of the control group (*P*<0.05). This indicates that the hemodynamic detection rate of POF patients is low, and the ovarian artery resistance is high. The ovarian artery parameters PI, RI, and S/D of the experimental group were significantly higher than those of the control group, and the differences were statistically significant (P<0.05). The higher the RI and PI, the higher the blood flow resistance, the worse the perfusion of the ovaries and the uterus, and the presence of blood supply disorders. It suggests that the blood flow resistance of POF patients is higher than that of normal people, and the ovarian and uterine perfusion is poor [29]. Because PI and RI are less affected by the acoustic beam and the cross-sectional area of blood vessels, ovarian artery parameters PI and RI can be used as specific indicators for evaluating POF.

## 5. Conclusion

In this work, 80 patients with idiopathic POF were selected as the experimental group, and 40 volunteers who underwent physical examination at the same period were selected as the blank control group. Transvaginal Doppler ultrasonography based on the improved Mean Shift algorithm was performed. Finally, it was proposed that transvaginal ultrasound based on the improved Mean Shift algorithm can clearly display the functional status and hemodynamics of patients' ovaries, and the ovarian artery parameters PI and RI can be used as specific indicators to evaluate premature ovarian failure. This study only evaluated the ovarian function status of patient before treatment, and did not examine their hemodynamics changes after treatment, lacking long-term data support. Later, it will collect the data of POF patients again to discuss the evaluation value of transvaginal color Doppler ultrasound in patients before and after treatment. In short, this study provided a data reference for the clinical application of color Doppler ultrasound in the diagnosis and treatment of POF patients.

## Figures and Tables

**Figure 1:** A: ultrasound image of premature failure; B: segmentation result of traditional mean shift algorithm.

**Figure 2:** Flow chart of improved mean shift algorithm.

**Figure 3:** Comparison on quantitative indicators of algorithm segmentation results. A, B, and C showed the comparison of RDD, ROD, and Dice, respectively. ∗ indicated that the difference compared with the algorithm in this study was statistically significant (*P*<0.05).

**Figure 4:** Ultrasound segmentation results of different algorithms. A was the original image; B was the segmentation result of the Snake model; C showed the segmentation result of the Live_wire algorithm; D showed the segmentation result of the traditional mean shift algorithm; and E was the segmentation result of the algorithm.

**Figure 5:** The general situation of patients in the experimental group and the control group. A showed the age, height, and weight of patients; B showed the hypertension, hyperlipidemia, and smoking history of patients.

**Figure 6:** Ultrasound data of a patient before and after treatment (24 years old, married). A was the transvaginal color Doppler ultrasound images before treatment; B showed the transvaginal color Doppler ultrasound images after treatment.

**Figure 7:** Comparison of ovarian size between experimental group and control group. ∗ indicated that the difference between the experimental group and the control group was statistically significant (*P*<0.05).

**Figure 8:** The hemodynamic detection rates of the experimental group and the control group. ∗ indicated that the difference between the experimental group and the control group was statistically significant (*P*<0.05).

**Figure 9:** Comparison of ovarian artery parameters between the experimental group and the control group. A showed the comparisons on EDV and PSV; B showed the comparisons on PI and RI; C was the comparison of S/D. ∗ indicated that the difference between the experimental group and the control group was statistically significant (*P*<0.05).

## Data Availability

The data used to support the findings of this study are available from the corresponding author upon request.
